The article "Let's Buy With Social Commerce Platforms Through Social Media Influencers: An Indian Consumer Perspective" was published in 2022. Journal: Front Psychol.

# Let's Buy With Social Commerce Platforms Through Social Media Influencers: An Indian Consumer Perspective

**DOI:** 10.3389/fpsyg.2022.853168

**Published:** 2022-04-15

**Authors:** Faizan Alam, Meng Tao, Eva Lahuerta-Otero, Zhao Feifei

**Affiliations:** ^1^School of Business Administrations, Dongbei University of Finance and Economics Dalian, Dalian, China; ^2^Universidad de Salamanca, IME, Salamanca, Spain

**Keywords:** social media influencers, s-commerce, trust, Indian s-commerce, COVID-19

## Abstract

The COVID-19 pandemic has had a substantial impact on the retail industry around the globe, including in the vast market of India. The response to the pandemic required stores to close and develop new ways to approach shoppers more efficiently. The worldwide usage of social media enabled the growth of social commerce (s-commerce). Influencers on s-commerce platforms use live broadcasting on their channels to promote endorsed products. The features of s-commerce influencers enhance users' trust in the online community and s-commerce intention, impacting their online purchasing intentions. In this study, we collected data from 379 Indian consumers to test the measurement and structural model using Partial Least Square-Structural Equation Modeling (PLS-SEM) to verify our conceptual framework. We found that trust in the online community and s-commerce intention are antecedents of online purchase intentions. Additionally, the results demonstrate that trust in Indian social media influencers and s-commerce intentions are vital for boosting consumers' purchase intention, verifying the hypothesized mediating effect of these factors. Based on these results, we suggest several managerial actions that could enhance the value of s-commerce for franchises, executives, e-retailers, and e-marketplaces.

## Introduction

Social commerce (s-commerce) is a subset of e-commerce that leverages social networking sites (e.g., Facebook, Instagram, YouTube, Twitter) and Web 2.0 technologies (Busalim, 2016; Hajli et al., 2017). Previous studies have defined s-commerce as the use of online technologies to allow people to interact through digital solutions and networks (Busalim, 2016; Lin et al., 2018). Social media platforms and discussion forums help online consumers to identify and buy products and services endorsed by social media influencers (SMI's) (Tao et al., 2020; Chin, 2021). In traditional e-commerce, consumers browse an electronic list of options before buying a product. Meanwhile, in s-commerce, consumers and sellers connect through social media networks to finalize their orders or trades (Cao et al., 2020). In 2020, s-commerce was expected to produce approximately USD 475 billion globally. From 2021 to 2028, the market is expected to grow by 28.4%, reaching roughly USD 3.37 trillion by 2028 (Statista, 2021). S-commerce in the Indian market represents an alternative to e-commerce. It enables swift communication and forms part of India's national transformation strategy, called Digital India or *Bharat* (KPMG Report, 2018). According to the India Brand Equity Foundation (IBEF), the Digital *Bharat* is optimistic about the growth of s-commerce (IBEF Report, 2021). The IBEF has projected that India's s-commerce market will be worth USD16–20 billion in 2025 and USD60–70 billion by 2030 (IBEF Report, 2021).

In India, there is a growing trend of promoting locally produced goods (Business Insider India Report, 2021). Due to logistics difficulties and nationwide shutdowns caused by the pandemic, online consumers have begun to purchase products with shorter shipping times (i.e., local goods from s-commerce providers). This has led domestic manufacturers to use SMI's to encourage consumers to purchase endorsed products and services through s-commerce (e.g., Bhattacharya, 2019; Droesch, 2019). India is home to the largest proportion of active Facebook, YouTube and Instagram users worldwide, with 410 million users on Facebook, 448 million users on YouTube, and 210 million users on Instagram (Statista-India Report, 2021). Few studies have examined the influence of SMI's on users' online shopping intention in s-commerce (e.g., Al-Nasser and Mahomed, 2020; Wang et al., 2020). The present study addressed the research gap concerning the impact of Indian SMIs' features (Todd and Melancon, 2018; Hou et al., 2020) on users' online purchasing intentions (Shaouf et al., 2016). It also examined users' trust in the community (Yahia et al., 2018) and s-commerce intention (Hajli, 2014). Previous studies have neglected the joint effects of trust in the community and social commerce intention on the link between SMI features and online purchase intentions in the Indian context. To the best of our knowledge, this is one of the few studies in including a model with these two effects to offer a comprehensive understanding of social commerce and users' shopping intentions, given the scarcity of studies in the Indian context. One of the most important advantages of social commerce is the social support to its members (hereunder through Indian SMIs) (Mo and Coulson, 2008; Oh and Syn, 2015), and taking this mind, our first research question also demonstrate how these influencers offer social support to their fans/followers. As a result of this engagement, influencers and online users have established trust in s-commerce. Successful online buying relationships are built on mutual trust, and trust is indeed a critical aspect in s-commerce activities (Hsu et al., 2014; Al-Debei et al., 2015). As a result of SMIs' suggestions, buyers are more likely to make purchases on social commerce platforms when they trust SMI's opinions.

Based on this, the study focused on two key research questions:

1. *How do SMIs demonstrate their characteristics and influence their fans to purchase endorsed goods?*
2. *What is the relationship between community trust, the intention to engage in s-commerce, and online purchasing intention?*

To answer these questions, we developed a model based on social presence theory. Our analysis explored important features of SMIs, including expertise (Todd and Melancon, 2018), attractiveness (Todd and Melancon, 2018), engagement (Todd and Melancon, 2018), and humor (Hou et al., 2020). We considered the association of these factors with consumers' online buying intentions. Trust and s-commerce intention are critical aspects of successful marketing campaigns on social shopping platforms (Lu et al., 2016). To test our assumptions, we surveyed 379 Indian social media users and analyzed the data using partial least square structural equation modeling (PLS-SEM).

This research makes several unique contributions. First, the study examined the position of Indian SMIs in the s-commerce market. Within the Indian economy, the Digital India strategy has played a significant role in persuading customers to make purchases online (KPMG Report, 2018). Thus, we examined the proactive antecedent of s-commerce and online shopping intention (Goraya et al., 2021), using social presence theory. Moreover, we considered the mediating role of community trust and s-commerce intention on the association between SMIs' features and users' online purchasing intentions. Previous studies have noted the role of online community behavior in relation to users' purchase of SMI-endorsed products from s-commerce platforms (Al-Nasser and Mahomed, 2020; Wang et al., 2020), and this research applies those concepts to the Indian context.

## Literature Review and Hypotheses

### Social Presence Theory

The conceptual framework for this study drew on social presence theory, which was developed by Short et al. (1976) and seeks to explain consumer s-commerce intentions. According to the theory, individuals' social presence on the Internet produces positive outcomes for the structure of society and improves their relationships with influencers (Short et al., 1976; Gunawardena, 1995). Social presence refers to the perceived availability of visual information-sharing in social interactions, compared to direct, vocal involvement. The availability of social presence is crucial to effective discussion between two or more individuals, which is aided by online technology (Kim et al., 2016). Furthermore, social presence is supported by online interactions, enabling consumer engagement on s-commerce platforms (Nadeem et al., 2020).

Online communication in s-commerce describes the extent to which an online social environment allows users to engage in truthful, cordial, intimate, and amicable interactions with one another (Zhang et al., 2014). This relationship is defined as the sense of closeness and friendliness that arises from conversing and socializing with other online users in a supervised context using online facilities (Yang et al., 2013; Fu et al., 2019). Such relationships drive consumers' attitudes, enabling them to create or maintain strong ties with influencers (Delbaere et al., 2021) and leading them to purchase endorsed products or services on s-commerce platforms.

### Social Media Influencers

Freberg et al. (2011) defined SMIs as “a novel sort of autonomous third-party endorser that influences community perspectives *via* posts, short videos, on social networks” (p. 90). SMIs are users who have achieved fame on social media through their knowledge and expertise on a particular subject. They cultivate enormous, passionate fanbases, encourage users to value their opinions, and motivate their audience to purchase endorsed products through frequent posts or livestreams. SMIs promote products or services on social media platforms such as Instagram, Facebook, Twitter, as well as through other media (Freberg et al., 2011). The content offered by SMIs is more interesting to consumers than traditional ads (Freberg et al., 2011). Thus, organizations are increasingly recruiting SMIs as brand ambassadors (Sudha and Sheena, 2017).

According to Freberg et al. (2011), the high level of engagement of SMIs' fans enables SMIs to convey their knowledge to online consumers and encourage them to purchase endorsed products. Consumer trust is another element that has evolved since the invention of the Internet (Johnson et al., 2018). SMIs have the power to persuade their followers and fans and establish trends on online platforms. Well-known SMIs have huge fanbases (Senft, 2013) and can make a considerable impression on their audiences, which increases their marketing value (Stever and Lawson, 2013).

#### Expertise, Attractiveness, Engagement, and Humor

SMIs have a favorable impact on their audience regarding s-commerce or e-commerce (Tao et al., 2020). SMIs use their expertise, attractiveness, engagement, and humor to provide information and educate their fans. One of the most important components of an influencer's reputation is their expertise, which refers to their level of familiarity with a given product. SMIs' attractiveness and engagement (i.e., their ability to effectively promote consumer viewership) can also contribute to their popularity. If an SMI possesses all these qualities, they can influence their fans' attitudes and behaviors, including their purchase intentions (Sokolova and Perez, 2021).

The accuracy and delivery of an influencer's knowledge or content are critical and can dramatically increase customer purchases (Haron et al., 2016), raising the value of goods and boosting community trust. Further, poor-quality social media posts are considerably more significant than creative and innovative content (Casaló and Ibáñez-Sánchez, 2018). As a result, attributes such as creativity, novelty, attractiveness, engagement, and humor are vital components of an influencer's personality (Todd and Melancon, 2018; Hou et al., 2020). Marketers often choose SMIs as ambassadors, relying on their knowledge, attractiveness, relationship with online shoppers, and brand or product fit. The influencer's socialization or reputation, which improves customer trust, is considered a critical criterion by both fans and advertisers. Customer interaction is enabled by the characteristics of particular s-commerce communities, which also serve as a framework for customer relationship management (Huang and Benyoucef, 2013; Ng, 2013). Customers can obtain more knowledge and build trust due to this social connection (Lin et al., 2017b). Based on these factors, we developed the following hypotheses:

*H1: The features of social media influencers are positively associated with users' trust in the community*.

*H2: The features of social media influencers are positively associated with users' social commerce intentions*.

### Trust in the Community

The e-commerce first transaction trust building model (TBM) was proposed by McKnight et al. (2002a). It highlighted how consumers build trust with SMI's and how it affects purchasers' behavior. We use the TBM model as a baseline foundation for this study's focusing on social commerce circumstances with a few improvements. Community trust is a significant topic in social media research (Hajli et al., 2017; Yahia et al., 2018). Users' trust in the community determines whether they believe information shared by other users. For instance, interacting with different users over a digital medium increases people's feeling of intimacy with the community (Goraya et al., 2021). According to researchers, trust is the readiness to be susceptible to the acts of individuals as they feel they are acting for their mutual benefit and will treat us favorably. In other words, we allow people to retain influence over us as we believe they will not harm us and might assist us in need time. Belief in the trustee's morality fosters trust in the business through trustor-to-trustee contact (hereunder SMI's and online community) (Morgan and Hunt, 1994; Wu et al., 2010). Information and knowledge regarding SMI-endorsed products validate consumers' willingness to trust other users (Lin et al., 2017a,b; Li and Ku, 2018), which may enhance their purchasing intentions. Previous research has identified a link between trust and online buying intentions (Ng, 2013; Shanmugam et al., 2016). Online users who contribute by giving their personal views and expertise through endorsements and suggestions on social media platforms are highly inclined to develop trust in online purchasing platforms (Kim and Park, 2013; Chen and Shen, 2015). Trust reflects the comprehensiveness of consumer interactions with their influencers, resulting in loyalty with SMI's. Individual social media users assure one another by exchanging knowledge, improving their trust and willingness to buy (Chen et al., 2016; Kim and Kim, 2018; Lin et al., 2018). Based on this, we developed the following hypotheses:

*H3: Trust in the community is positively associated with online purchasing intention*.

*H4: Trust in the community is positively associated with social commerce intentions*.

### Social Commence Intention

Intention is a common assessment adopted by behavioral academics to estimate potential individual behavior (Sheikh et al., 2019). Behavioral intention is closely connected to actual behavior (Chen et al., 2018; Wang et al., 2020). The primary goal of s-commence is to capitalize on interactions on a social network to increase economic returns (Liang and Turban, 2011). In s-commerce, intention refers to an action that a current and future purchaser intends to perform or a behavior they are expected to engage in Shin (2013). S-commence can lead to economic advantages such as increased consumer retention or revenue (Lin et al., 2017a). In today's Internet-based society, both influencers and users have a strong desire to purchase and spread trade information using s-commerce platforms. This is referred to as the s-commence intention (Chen and Shen, 2015). Users may form a social connection to obtain further benefits (Yang et al., 2015), and this can create several personal interactions from which such users gain knowledge (Razak et al., 2016). Through s-commerce networks, influencers interact with their friends and broader social circle. For example, they give feedback regarding products or services they have purchased and experienced. Based on this notion, we proposed the following hypothesis:

*H5: Social commerce intentions are positively associated with online purchasing intention*.

### Online Purchasing Intention

According to Spears and Singh (2004), purchasing intention indicates “a person's deliberate goal to buy a specific product” (p. 56). De Magistris and Gracia (2008) argued that purchasing intention anticipates practical buying behavior, indicating that purchasers may be ready to acquire a specific product. Purchase intention is considered an essential element in determining buying behavior (Shin and Biocca, 2017; Shin and Hwang, 2017). It refers to the intention expressed by customers regarding their desire to buy a product or service based on personal choices and their overall assessments (Pang, 2021). According to Ko and Megehee (2012), buying inclinations are purchasers' behavioral intention to buy a product or service. Furthermore, Sokolova and Perez (2021) suggested that online experience with SMIs increases fans' purchasing intentions due to the fans' trust in their idols. New technologies and the emergence of the Internet have led to a diversity of business associations and sales, leading to research examining online purchasing intentions in s-commerce (Zhang and Wang, 2021). Customers in s-commerce anticipate, investigate, and attentively consider their options when purchasing a product. However, SMIs significantly impact consumers' purchasing intentions *via* their suggestions and assessments (Meilatinova, 2021).

### Mediation Role of Trust in the Community and Social Commerce Intention

It is well-established that trust leads to an enhancement in members' eagerness to use and share knowledge on websites, which is demonstrated by earlier findings (e.g., McKnight et al., 2002a,b; Wu and Tsang, 2008). For example, in the s-commerce context, increasing consumer trust enhances customers' willingness to make online purchases (Wu and Tsang, 2008; Harrigan et al., 2021; Tao et al., 2021). To a greater extent, consumers' willingness to buy from influencers might increase their trust in SMIs. Therefore, online communities establish trust in SMIs and are more likely to engage in online purchasing transactions (Zhou et al., 2021a). In the light of this, we propose the following hypothesis:

*H6: Trust in the community mediates the association between features of social media influencers and online purchasing intention (**Figure 1**)*.

**Figure 1:** Conceptual framework.

Online users are increasingly more concerned with e-business content. In the s-commerce context, sharing and interaction are the foremost for individuals. Individuals that engage in s-commerce attribute close attention to receiving valuable content and reaching better buying behavior (Liang et al., 2011; Kim, 2013; Hu et al., 2022). Therefore, such requirements should be enough if successful social relationships enable knowledge sharing among online communities (Kusumasondjaja, 2017). With regular social encounters with SMI's, knowledge can be more easily transferred from origin to destination. As a result, an e-commerce platform's degree of social commerce intention becomes critical toward its ability to enhance individuals' buying behavior (Hu et al., 2022). We hypothesize accordingly:

*H7: social commerce intention mediates the association between features of social media influencers and online purchasing intention*.

## Research Methodology

This study was conducted in India and involved a survey of 379 Indian research participants (of a total of 420 questionnaires). All the participants regularly purchased goods on s-commerce platforms based on SMIs' opinions. To select the SMIs for this study, we randomly selected 30 Indian volunteers who were familiar with SMIs and active on social media platforms. We asked them to suggest well-known Indian SMIs of both genders (Pornpitakpan, 2004). As shown in Table 1, we used the suggestions to develop a list of 12 Indian SMIs (six male and six female) and divided them into three categories: (1) fashion, beauty and travel, (2) food, and (3) general. This ensured that the participants were familiar with the SMIs. Our target for the study was to collect data from large s-commerce platforms such as Instagram, Facebook, and YouTube, as those platforms represent a significant portion of Indian SMIs and their followers. Thus, we targeted users of those platforms. We used non-probability criterion-based convenience sampling, as suggested by Brus and De Gruijter (2003). The survey was first published in English to a pilot sample of 30 respondents and five senior professors, then revised based on their feedback. The data was gathered between June and September of 2021. We uploaded and distributed the questionnaire using Microsoft Forms, an online survey platform. Before the respondents started the questionnaire, they were provided with instructions that ensured their privacy and described the objectives of the research.

**Table 1:** Numbers of followers of Indian social media influencers.

**Category**	**Instagram**	**Facebook**	**You Tube**
**Fashion, beauty, and travel influencers**			
Masoom Minawala Mehta	1.1 M	205 K	52 K
Komal Pandey	1.5 M	35.6 K	991 K
Abhi and Niyu	2.2 M	1.5 M	2.01 M
Aakriti Rana	818 K	15.7 K	154 K
Prajakta Koli	4.5 M	1.2 M	6.45 M
**General influencers**			
Ajay Nagar	14.2 M	2.3 M	33.6 M
Amit Bhadana	5.5 M	9.2 M	23.6 M
Ankur Warikoo	1.0 M	366 K	1.2 M
Kusha Kapila	2.1 M	16 K	304 K
Mohena Kumari Singh	1.1 M	–	591 K
**Food and fitness influencers**			
Karan Dua	953 K	105 K	1.79 M
Ranbeer Allahbadia	1.7 M	13 K	2.88 M

*Source: Influencers social media accounts (23 December 2021).

### Sample Profile

All the participants were Indian nationals, of which 49% were male, 42% were female, and 9% preferred not to say. In terms of age, 11% of the participants were <20 years old, 44% were aged between 21 and 30, 18% were between 31 and 40, 11% were between 41 and 50, and 16% were over 50 years old. Concerning education, 12% had a high school diploma or below, 53% held a bachelor's degree, 22% had postgraduate qualifications, and 13% had a doctorate. One-third (33%) of the participants were employed, 39% were self-employed, 22% were unemployed, and the remaining 6% preferred not to say. Most (65%) of the participants were unmarried, 24% were married, and 11% were divorced. The largest proportion (37%) of the participants were Hindu, 19% were Muslim, 17% were Sikh, 16% were Christian, and the remaining 11% were from other religious communities. Table 2 summarizes the participants' characteristics.

**Table 2:** Demographic profile of respondents.

**Demographics**	**Category**	**Frequency**	**Percent**
Gender	Male	186	49
	Female	159	42
	Preferred not to say	34	9
Age	Below 20	42	11
	21–30	165	44
	31–40	70	18
	41–50	40	11
	Above 50	62	16
Education	High school or below	44	12
	Bachelors	202	53
	Masters	83	22
	PhD	50	13
Occupation	Employed	125	33
	Self-employed	148	39
	Unemployed	83	22
	Preferred not to say	23	6
Marital status	Unmarried	248	65
	Married	91	24
	Divorced	40	11
Religion	Hindu	138	37
	Muslim	74	19
	Sikh	68	17
	Christian	59	16
	Others	40	11

### Construct Measurement

The survey used a 5-point Likert scale, with the responses ranging from “Strongly disagree” (rated as 1) to “Strongly agree” (rated as 5). The research items were drawn from the literature and adapted to the framework of this research. The features of SMIs were measured across four dimensions: expertise, attractiveness, engagement (Todd and Melancon, 2018), and humor (Hou et al., 2020). We also measured trust in the community (Yahia et al., 2018), s-commerce intentions (Hajli et al., 2017), and online purchase intentions (Shaouf et al., 2016). Table 3 shows the research constructs and their items. We used SmartPLS v.3.2.7 to conduct the PLS-SEM test (Mateos-Aparicio, 2011).

**Table 3:** Constructs, reliabilities, validities, and variance inflation factor.

**Constructs**	**FL**	**α**	**rho_A**	**CR**	**AVE**	**VIF**
**Features of social media influencers**		**0.878**	**0.883**	**0.917**	**0.734**	
**Social media influencers expertise**		0.928	0.928	0.965	0.933	
This social media influencer is knowledgeable.	0.966					3.987
This social media influencer is a good teacher.	0.966					3.987
**Social media influencers attractiveness**		**0.867**	**0.868**	**0.938**	**0.883**	
This social media influencer is attractive.	0.941					2.419
This social media influencer is charming.	0.938					2.419
**Social media influencers engagement**		**2.419**	**2.419**	**2.419**	**2.419**	
This social media influencer is fun to watch.	0.881					2.172
This social media influencer is entertaining.	0.898					2.486
This social media influencer is enjoyable to watch.	0.902					2.456
**Social media influencers humor**		**0.867**	**0.867**	**0.919**	**0.79**	
This social media influencer is funny.	0.867					1.988
This social media influencer is humorous.	0.892					2.408
This social media influencer is amusing.	0.907					2.650
**Trust in the community**		**0.921**	**0.922**	**0.944**	**0.809**	
I trust in the information provided by the other community members.	0.905					3.284
I trust in the community members to be honest.	0.901					3.351
I trust the community members to be trustworthy.	0.937					4.447
I do not trust that the community members will take advantage of me.	0.854					2.409
**Social commerce intentions**		**0.911**	**0.912**	**0.944**	**0.849**	
I am willing to accept experiences and suggestions from social media influencer about endorsed products.	0.911					2.937
I am willing to buy the products recommended by the social media influencer.	0.940					3.815
I will consider my social media influencer shopping experiences when I want to shop.	0.914					2.917
**Online purchase intentions**		**0.907**	**0.913**	**0.941**	**0.842**	
I am interested in making the purchase from social commerce platforms.	0.922					3.115
I am willing to purchase the product from social commerce platforms.	0.924					2.904
I will probably purchase the product from social commerce platforms.	0.907					2.879

*FL, Factor loadings; α, Cronbach alpha; CR, Composite reliability; AVE, Average variance extracted; VIF, Variance inflation factor. Bold values mean constructs where non bold values mean items that form the construct*.

### Analysis

We filtered the data before conducting our analysis to verify its accuracy and evaluate the normality of the target variable. First, the missing values were inserted using the average of the relevant subscale. Secondly, we scrutinized the dataset for outliers, meaning values larger than 3.5 standard deviations from the sample mean (Hair et al., 2013). Thirdly, we used SmartPLS to analyze the data using PLS (Ringle et al., 2015). Finally, we used 5,000 sample sizes of a consistent PLS bootstrapping approach with replacement to evaluate the empirical validity of the measurement estimations. We also ran a PLS multi-group analysis (PLS-MGA) to determine whether the model subgroup parameter estimates differed significantly (Sarstedt et al., 2011).

### Measurement Model

#### Common Method Bias

We checked for common method bias (CMB) because the current study predictor variables were represented by a similar responding method (Podsakoff et al., 2003). Previous studies (Schwarz et al., 2017; Rodríguez-Ardura and Meseguer-Artola, 2020; Kock et al., 2021) have proposed various precautions to regulate CMB, such as ensuring participant anonymity, avoiding ambiguous research questions, and offering detailed guidance to reduce bias and errors. We used a more modern approach and evaluated CMB by analyzing the collinear constructs and associated items (Rodríguez-Ardura and Meseguer-Artola, 2020). First, we measured the associated items variance inflation factor (VIF). As shown in Table 3, we found that the VIF values were <5, suggesting that CMB was not an issue. Checking that inter-construct correlation is below 0.90 is another way to test for CMB (Bagozzi et al., 1991). As shown in Table 4, the results in this study passed that test. Thus, this analysis met the Fornell and Larcker (1981a) criteria for confirming discriminant validity. Hence, CMB was not an issue in the testing of the structural model.

**Table 4:** Discriminant validities, *R*^2^, *Q*^2^, *f*^2^ and model fit.

**Constructs**	**OPI**	**SMIAS**	**SMIEG**	**SMIET**	**SMIHR**	**SCI**	**TCI**
**(Fornell Larker)**							
OPI	0.918						
SMIAS	0.672	0.94					
SMIEG	0.642	0.793	0.894				
SMIET	0.599	0.688	0.688	0.966			
SMIHR	0.68	0.548	0.576	0.566	0.889		
SCI	0.697	0.672	0.66	0.736	0.597	0.922	
TCI	0.707	0.633	0.642	0.712	0.602	0.839	0.900
**(HTMT method)**							
OPI							
SMIAS	0.755						
SMIEG	0.719	0.881					
SMIET	0.651	0.766	0.763				
SMIHR	0.765	0.631	0.661	0.631			
SCI	0.763	0.756	0.739	0.801	0.672		
TCI	0.77	0.708	0.715	0.771	0.674	0.824	
**Constructs**	**TCI**	**SCI**	**OPI**	**model fit**			
***R** ^**2**^*	0.574	0.752	0.534				
***Q* ^2^**	0.437	0.604	0.424				
***f* ^2^**							
FSMI	1.352	0.200					
SCI	0.078						
TCI	0.580	0.110					
SRMR	0.050						
NFI	0.895						
GOF	0.636						

*OPI, Online purchase intentions; SMIAS, Social media influencers attractiveness; SMIEG, Social media influencers engagement; SMIET, Social media influencers expertise; SMIHR, Social media influencers humor; SCI, Social commerce intentions; TCI, Trust in the community; FSMI, Features of social media influencers*.

#### Internal Consistency

Cronbach's alpha and composite reliability (CR) are the key measurements of internal consistency. Hair et al. (2016) suggested that the value of Cronbach's alpha should be between 0.60 and 0.70. As shown in Table 3, Cronbach's alpha in the current study ranged from 0.87 to 0.92, which was acceptable. CR refers to the internal consistency of modified items conferring to precise variables (Henseler et al., 2009). The minimum permissible value of CR is 0.60 (Fornell and Larcker, 1981a). As shown in Table 3, the internal consistency of the variables varied from 0.917 to 0.944, meaning that the CR exceeded the required value.

#### Construct Validity

Content validity, convergent validity, and discriminant validity are all measured using latent variables (Fornell and Larcker, 1981b; Hair et al., 1998; Chin et al., 2003). Discriminant validity is demonstrated when the average variance extract (AVE) square root is higher than the actual inter-item associations, as shown in Table 4. Moreover, Table 3 displays the permissible ranges and results for AVE, Cronbach's alpha, and composite reliability.

### Structural Model

In this study, the standardized root mean residual (SRMR) was 0.05. A value lower than 0.1 indicates a strong model fit (Hu et al., 1998; Henseler et al., 2014). Values for the normed fit index (NFI) range from 0 to 1, with values closer to 1 indicating a better fit. NFI values >0.9 are considered appropriate (Lohmöller, 1990). As shown in Table 3, the model's NFI was 0.89, indicating an excellent fit. We also calculated the goodness of fit (GOF) value, as given by Tenenhaus et al. (2005), to assess the overall validity of the model. The GOF value was 0.63, exceeding the minimum value of 0.360 (Wetzels et al., 2009).

#### Coefficient of Determination (R^2^), Effect Size (f^2^), Predictive Analytics Q^2^

*R*^2^ values of 0.75, 0.50, and 0.25 are characterized as substantial, moderate, and weak, respectively (Henseler et al., 2016; Sarstedt et al., 2017). In this study, the *R*^2^ values for trust in community and influencers, s-commerce intentions, and online purchasing intentions were 0.57, 0.75, and 0.53. Rather than depending only on *R*^2^, some scholars have suggested the Stone-Geisser *Q*^2^ as a potentially effective determinant of a model's predicted relevance (Sarstedt et al., 2017). *Q*^2^ is calculated using the blindfolding technique; it determines whether the path model accurately predicts the actual value. *Q*^2^ values of 0.02, 0.15, and 0.35 indicate low, medium, and considerable predictive significance (Sarstedt et al., 2017). In our model, the *Q*^2^ values for trust in community and influencers, s-commerce intentions, and online purchasing intentions were 0.43, 0.60, and 0.42, indicating strong predictive relevance. Finally, we evaluated the effect size (*f*^2^). The *f*^2^ measurement is used to estimate the latent variable relevance over each endogenous variable. *f*^2^ values of 0.02, 0.15, and 0.35 indicate small, medium, and large effect sizes (Cohen, 1988). As shown in Table 4, the *f*^2^ values for our model were acceptable.

#### Hypothesis Testing

The path coefficients (β), T statistics (*t*), and significance (*p*) values were measured in the structural model. Using this model, we tested the acceptance or rejection of the hypotheses based on the results. As shown in Table 5, we found that the features of SMIs have a positive effect on trust in the community (β = 0.841, *t* = 35.920, *p* < 0.001) and a positive effect on s-commerce intentions (β = 0.346, *t* = 4.539, *p* < 0.001). Trust in the community has a positive effect on online purchasing intentions (β = 0.443, *t* = 3.455, *p* < 0.01) and on s-commerce intentions (β = 0.624, t = 8.173, *p* < 0.001). S-commerce intentions have a positive effect on online purchasing intentions (β = 0.358, *t* = 2.781 *p* < 0.01). Thus, hypotheses H1, H2, H3, H4, and H5 were supported (Figure 2).

**Table 5:** Model results.

**Relationship**		**Beta (β)**	***T* value**	***P*-value**	**Decision**
**Direct effects of constructs**				
H1	FSMI → TCI	0.841	35.920	0.000	Supported
H2	FSMI → SCI	0.346	4.539	0.000	Supported
H3	TCI → OPI	0.443	3.445	0.001	Supported
H4	TCI → SCI	0.624	8.173	0.000	Supported
H5	SCI → OPI	0.358	2.781	0.006	Supported
**Mediating effects of TCF and SPI**				
H6	FSMI -> TCI -> OPI	0.372	3.359	0.001	Supported
H7	FSMI -> SCI -> OPI	0.124	2.169	0.031	Supported

*FSMI, Features of social media influencers; TCI, Trust in the community; SCI, Social commerce intentions; OPI, Online purchase intentions*.

**Figure 2:** Path analysis.

We found that the features of SMIs have a direct effect on online purchasing intention (β = 0.478, t = 8.015, *p* < 0.001), and trust in the community mediates the positive relationship between the features of SMIs and online purchasing intentions (β = 0.372, t = 3.359, *p* < 0.01), supporting hypothesis H6. S-commerce intentions also mediated this relationship (β = 0.124, t = 2.169, *p* < 0.05), supporting hypothesis H7. We found complementary partial mediation existed based on the results and Zhao et al. (2010) recommendation. As Zhao et al. (2010) suggested, partial mediation existed if the direct effect and mediation effect were positive. So based on this recommendation, we can say partially mediation existed. Complementary partial mediation is often called a “positive confounding” or a “consistent” model (Zhao et al., 2010).

## Conclusion

The purpose of this research was to investigate the involvement of SMIs in s-commerce and the overall mediating impact of community trust on s-commerce intentions and behavior (i.e., online purchasing intentions) in India (Hajli, 2013). We developed a conceptual framework centered on social presence theory and proposed seven hypotheses. Our results validate these hypotheses, indicating a positive connection between the features of SMIs, trust in the community, and s-commerce intentions. The findings are also consistent with theories of s-commerce, which claim that the behavior of internet users is affected by the actions of SMIs (Horne et al., 2017).

As stated above, our findings confirm the positive association between the features of SMIs, trust in the community, and s-commerce intentions. This suggests that SMIs' traits influence the behavior of their fans, followers, and other users, resulting in increased community trust and s-commerce intentions (Hajli, 2013, 2014; Kong et al., 2020). Furthermore, the results suggest that trust in the community and SMIs are positively correlated with s-commerce intentions and online purchasing intentions, indicating that online consumers prefer s-commerce sites over e-commerce platforms (Lu et al., 2010, 2016; Ng, 2013). Finally, the results demonstrate a favorable association between s-commerce intentions and online purchasing intentions, indicating that online consumers are likely to purchase products endorsed by SMIs. This proves the validity of the current research.

This study also demonstrates the mediating function of trust in the online community and s-commerce intentions on the relationship between the features of SMIs and online purchase intentions, based on social presence theory and prior s-commerce studies. Thus, s-commerce platforms can establish valuable trade relationships with SMIs, who offer users awareness and empathy. This integration may arouse the curiosity of customers looking for relevant information to purchase or exchange (Zhou et al., 2021b). As a result, consumers who deeply trust s-commerce sites are more interested in online shopping *via* SMIs and in promoting their overall knowledge (Hajli, 2019).

The first research question for this study asked, “How do SMIs demonstrate their features and influence their followers to acquire recommended goods?.” We found that SMI characteristics have an impact on user behavior in online communities. The adoption of SMI marketing by brands improves community trust and s-commerce intentions, resulting in increased s-commerce earnings (Yusuf and Busalim, 2018). Customers in India are suspicious of e-commerce platforms due to fraud (Chawla and Kumar, 2021). S-commerce platforms, in contrast, provide users with an assurance of trust and a supportive atmosphere (Soleimani, 2021). As a result, employing Indian SMIs could be a useful way for brands to convey information, raise users' exposure to their products, strengthen trust, and increase sales. Influencers can help businesses to build personal contacts with and provide information to their prospective customers (Nosi et al., 2021).

The second key research question focused on the relationship between community trust and the intention to interact in s-commerce, as well as online purchasing intention. Our results show that buyer trust is among the most important variables in ensuring consumer continuity and loyalty to particular SMIs. Consumers may quickly change platforms or influencers if they are dissatisfied with a particular SMI (Gulamali and Persson, 2017). Thus, customer purchase decisions are influenced by their trust in the community and particular influencers; the long-lasting performance of interactions promotes users' s-commerce intentions.

### Theoretical Implications

This research generated significant theoretical insights into s-commerce and SMIs. For instance, the results show that SMIs are a multidimensional second-order construct with four first-order indications: expertise, attractiveness, engagement, and humor. The empirical literature concerning the second variable suggests that the characteristics listed above reflect the overall complexity of SMIs. Thus, it is critical to consider potential factors beyond users' colleagues, relatives, and friends, including individuals who are part of the same shared community. First, although live-streaming by SMIs is gradually being linked to s-commerce, few studies have considered the impact of SMIs' features on this new form of consumption. Existing studies on the potential of social presence theory in online s-commerce environments (Lu et al., 2016; Hajli et al., 2017) explore the existing framework and extend the current theory.

Moreover, we also include the mediation effect of trust in the community and social commerce intention with the association of features of SMI's and online purchasing intention. Due to the expected prominence of interaction features in social commerce, it is worth considering what can anticipate a better relationship with SMI's and online users. The characteristics of influencers also significantly affect s-commerce intention, demonstrating the value of social presence theory in the context of s-commerce platforms. Previous research has found that SMIs can influence consumer behavior and purchase intent by fostering trust (Hajli, 2015; Lu et al., 2016). The current study incorporated influencers' attributes and users' online purchase intention into the model. Online purchase intention is explained by the mediating role of community trust and s-commerce intention, validating the role of social presence theory in the proposed framework. Thus, this research extends the use of social presence theory in the context of s-commerce intention. This is valuable if, for example, a brand is seeking to spread knowledge about SMI-endorsed products to establish social relationships (James et al., 2015). Importantly, this study was based on buyers' social relationships, as a social business is defined by customers' intended and unintended communications.

### Managerial Implications

Our findings are particularly useful to marketing specialists and managers tasked with maximizing the marketing potential of influencers through strategic plans and tools. According to Sun and Xu (2019), if SMIs successfully build connections with their consumers, they can substantially impact all elements of consumer buying behavior. For example, most online consumers have been exposed to fraudulent sellers in online transactions (Bhattacharjee and Goel, 2005). This has caused low levels of consumer trust regarding online purchases. Our results suggest that trust in the community and s-commerce intentions might help to address this problem by creating a pleasant shopping environment and increasing users' online buying intentions.

Thus, this research creates opportunities for retailers to maximize the impacts of s-commerce on purchase intention and sales. The ability of SMIs to broadcast information has significantly improved (Zhang et al., 2020; Jodén and Strandell, 2021), meaning that consumers perceive SMI-endorsed product information as more trustworthy than information from official advertisements (Sohaib, 2021). The popularity of s-commerce platforms produces beneficial interactions for online users and significantly impacts their online purchase intentions. Accordingly, with the support of the current research framework, e-retailers should leverage SMIs to achieve economic benefits on s-commerce platforms.

Our research also shows that trust and s-commerce intention can raise consumers' willingness to purchase goods. Users may modify their pre-existing purchase goals due to the credible suggestions of influencers they admire (Hudders et al., 2021). Online social media platforms that specialize in s-commerce (e.g., Facebook, Instagram, and YouTube) offer a larger ecosystem for their customers and influencers. Thus, s-commerce marketers should focus on establishing a pleasant atmosphere and should hire influencers based on their target dialects and regions. The framework described in this study, for example, clearly indicates that young innovators in India should leverage social media sites in their marketing, as such sites have lower operational costs and larger and more diverse potential audiences. They also enable more personal customer care. Such measures will help young innovators to grow their businesses. This will contribute to the “Made in India” campaign, which supports the goals of young Indians.

### Limitations and Future Research Lines

This study had some limitations, which should be addressed in future research. First, we used snowball sampling to obtain data from the North Capital region of India, limiting the territorial scope of the study. In future studies, the framework developed in this study could be applied to different Indian provinces to better understand online buying behavior on social networking websites *via* SMIs. Furthermore, our approach could be applied to other highly digitalized Asian nations, where many users have access to shopping platforms (Ahmed et al., 2017; Xu et al., 2021). Secondly, factors such as electronic word of mouth, the trustworthiness of information, and information-seeking were not included in our framework. Future research could investigate the impact of these parameters on consumers' online buying intentions. Thirdly, future studies could investigate the impact of Indian SMIs' endorsements on foreign residents' online purchasing intentions (Yu et al., 2018). India's influencers have a huge impact on users in Western countries. Thus, future research could explore the role of factors such as repeat purchase intentions and online satisfaction in developing long-term interactions with both Indian and foreign audiences *via* SMIs.

## Data Availability Statement

The raw data supporting the conclusions of this article will be made available by the authors, without undue reservation.

## Author Contributions

Study conception, design, data collection, analysis, and interpretation of results by FA. ZF and MT draft manuscript reviewing, editing, and supervision by MT and EL-O. All authors reviewed the results and approved the final version of the manuscript. All authors contributed to the article and approved the submitted version.

## Funding

The authors thank the Spanish Ministry of Science and Innovation (PID2020-113469GB-I00), the Junta de Castilla y León and the European Regional Development Fund (Grant CLU-2019-03) for the financial support to the Research Unit of Excellence Economic Management for Sustainability (GECOS) and the National Natural Science Foundation of China (中国国家自然科学基金项目) (Grant No. 项目批准号: 72072026).

## Conflict of Interest

The authors declare that the research was conducted in the absence of any commercial or financial relationships that could be construed as a potential conflict of interest.

## Publisher's Note

All claims expressed in this article are solely those of the authors and do not necessarily represent those of their affiliated organizations, or those of the publisher, the editors and the reviewers. Any product that may be evaluated in this article, or claim that may be made by its manufacturer, is not guaranteed or endorsed by the publisher.
